This article has been retracted.

# All-Trans Retinoic Acid Enhances Chemosensitivity to 5-FU by Targeting miR-378c/E2F7 Axis in Colorectal Cancer

**DOI:** 10.1155/2021/5338934

**Published:** 2021-07-19

**Authors:** Ji Li, Qing Xiang, Mei Wang, Hongchang Zhang, Rong Liang

**Affiliations:** ^1^Department of Pharmacy, Qilu Hospital (Qingdao), Cheeloo College of Medicine, Shandong University, Qingdao, Shandong 266035, China; ^2^Department of Emergency, Rizhao Hospital of TCM, Rizhao 276800, China; ^3^PIVAS, Qingdao Central Hospital Affiliated to Qingdao University, Qingdao 266000, China; ^4^Infectious Diseases Department, Zhangqiu District People's Hospital, Jinan 250200, China; ^5^Department of Proctology(II), Qilu Hospital (Qingdao), Cheeloo College of Medicine, Shandong University, Qingdao 266035, Shandong, China

## Abstract

Colorectal carcinoma (CRC), a life-threatening malignancy, has been found to present resistance to 5-fluorouracil (5-FU) and cause a poor prognosis for patients. Previous studies have proved that all-trans retinoic acid (ATRA) could inhibit the development of CRC cells. In addition, miR-378c was discovered to exert a vital role in various cancers. In this study, we utilized MTT (3-(4,5-dimethylthiazol-2-yl)-2,5-diphenyltetrazolium bromide), transwell assay, and flow cytometry to confirm that ATRA was able to enhance the inhibitory effects of 5-FU on HCT116 cells effectively by promoting cell apoptosis. Then, ENCORI database (http://starbase.sysu.edu.cn/) was employed to predict that miR-378c was downregulated dramatically in CRC and E2F7 was the direct target of miR-378c. QRT-PCR (quantitative real-time polymerase chain reaction) was conducted to verify that the expression level of miR-378c was decreased while E2F7 expression was upregulated in CRC tissues compared with para-carcinoma tissues. Additionally, treatment of 5-FU combined with ATRA could increase miR-378c expression, whereas it decreased the expression of E2F7. Dual-Luciferase Reporter assay results revealed that miR-378c could regulate the load of E2F7 by binding to its 3′UTR directly. Furthermore, miR-378c inhibitor or vector with E2F7 partially counteracted the effects of 5-FU combined with ATRA on viability, migration, invasion, and apoptosis of HCT116 cells. In conclusion, our study aims to confirm that ATRA enhances chemosensitivity to 5-FU of patients with CRC and expound the potential molecular mechanisms.

## 1. Introduction

Increasing developments had been made in treating CRC recently. However, CRC remains the second main reason for death associated with tumors and is graded as the fourth diagnosed malignancy worldwide [1–3]. Chemotherapies were the foundation of treatment for patients with CRC in recent decades even though they exhibited obvious toxicity in addition to being ineffective [4]. Due to the limitations of early symptoms as well as screening technologies, many patients with CRC are diagnosed at the advanced stage [5]. The reason that contributes to poor results for patients is mainly recurrence in addition to metastasis of CRC [6]. Over the past few decades, the useful therapy for patients with CRC is the chemotherapy based on fluorouracil. Nevertheless, patients are becoming more and more resistant to 5-FU, which is the major barrier for treating effectively [7, 8]. Therefore, multiple anticancer agents are employed to combine with 5-FU to enhance therapeutic effectiveness for CRC at present [9]. ATRA, one of the important metabolites of vitamin A, has great potential to prevent and treat cancer [10]. ATRA plays promising roles in various cancers including breast cancer, glioblastoma, and head-and-neck cancer [11, 12]. Additionally, Yang et al. found that ATRA is able to inhibit colon cancer cells from proliferating via mediating sponge miR3666 [11]. María Ángeles Castro et al. primarily revealed that retinoids and 5-FU have synergistic effects on Caco-2 cells [13]. However, the detailed functions and mechanisms underlying 5-FU in addition to ATRA are uncovered now.

MicroRNAs, as the endogenous, non-coding RNAs, have the ability to regulate target genes, and a variety of witnesses have testified that microRNAs are correlated to the progression of various cancers [14–16]. MicroRNAs can serve as either cancer suppressor genes or oncogenes to affect the proliferation, migration, and therapy of cancers [17]. A load of certain genes related to metabolism, stress responses, and cell apoptosis will be regulated by the aberrant transcription of specific miRNAs [18, 19]. Take miR-433, for example; it decreases resistance of cervical cancer cells to 5-FU through regulating the expression of TYMS [20]. Mir-20313, in addition to miR-197, could regulate the reactivity of colorectal cells to 5-FU by changing TYMS expression [21, 22]. MiR-378c belonging to the miR-378 family has been found to have a close relationship with cancers. For example, miR-378c is decreased in gastric cancer tissues, according to previous reports [23]. Furthermore, we consulted the database and found that miR-378c was downregulated significantly in COAD (colon adenocarcinoma), but its effects on CRC are unclear.

Therefore, our study reveals the functions and detailed molecular mechanisms of ATRA combined with 5-FU for CRC via the miR-378c/E2F7 axis.

## 2. Materials and Methods

### 2.1. Patients and Tissue Samples

CRC and para-carcinoma tissues were extracted from 15 patients diagnosed with early CRC and treated with radical surgery at Qilu Hospital, Jinan, Shandong, China. In addition, no patients were treated systematically before surgery. All patients provided written informed consent. The isolated tissues were put in liquid nitrogen immediately. All experiments involved in this study were in accordance with the ethics committee of the Qilu Hospital, Jinan, Shandong, China.

### 2.2. Cell Culture

The HCT116 cell line was purchased from COBIOER in Nanjing and was cultured with McCoy's 5A (Gibco, USA), including 10% FBS (fetal bovine serum) at 37°C.

### 2.3. Cell Treatment

Different concentrations of 5-FU and ATRA were dissolved in dimethylsulfoxide (DMSO, Thermofisher) solution. HCT116 cells were cultured overnight and treated with the indicated concentration of 5-FU in addition to ATRA for 24 hours. Additionally, the control group referred to DMSO solution with the same volume.

### 2.4. Cell Transfection

HCT116 cells (1 × 10^5^ cells/well) were planted in specific well plates. Indicated mimic, inhibitor, or vector was transfected into HCT116 cells when cells reached 70% confluence with Lipofectamine 3000 (Thermofisher, USA). After culturing for 24 hours, HCT116 cells were collected for the following assay.

### 2.5. MTT Assay

HCT116 cells (1 × 10^3^ cells/well) were planted in a 96-well plate and cultured for a night. Then, different doses of 5-FU and ATRA were used to treat HCT116 cells which have been transfected with indicated vectors. After 24 hours, 0.5 mg/ml MTT was added into every well for 4 hours. Finally, the OD value at 550 nm was recorded with a Flash reader (Thermofisher, USA) to represent cell viability.

### 2.6. Cell Apoptosis

HCT116 cells were planted in 6-well plate overnight. Then, different doses of 5-FU and ATRA were used to treat HCT116 cells which were transfected with indicated vectors. After 24 hours, all cells were obtained in HEPES buffer (119.15 g HEPES (4-hydroxyethyl piperazine ethanesulfonic acid), 0.5–1 M NaOH, PH 6.8–8.2, capacity to 500 ml), and the mixture was centrifuged to abandon supernatant. Next, cells were stained by Annexin V/PI for half hour. Subsequently, flow cytometry was conducted to analyse cell apoptosis rate by using CellQuest software (Becton, USA). The four quadrants represent normal (third quartile), early apoptosis (second quartile), late apoptosis (fourth quartile), and necrotic (first quartile) cells.

### 2.7. Transwell Assay

For migration assay, HCT116 cells (5 × 10^4^ cells) in serum-free medium were planted in the upper transwell chamber containing an insert (8-mm pore; Corning, USA). Nevertheless, cells were seeded in the upper transwell chamber containing an insert prepared with Matrigel. Medium with 10% FBS as the chemoattractant was placed in the lower transwell chamber. After 24 hours, cells still staying on the upper part were cleared away by using cotton wool; however, cells migrating or invading to the lower chamber were fixed, stained, and recorded with an inverted microscope (Olympus, Japan).

### 2.8. Dual-Luciferase Reporter Assay

The sequence of E2F7-WT or E2F7-MUT was amplified and constructed into pGL3 plasmid (Thermofisher, USA). Specific mimic or vector was transfected into HCT116 cells by Lipofectamine 3000. After 36–72 hours, a microplate reader was used to measure and record the luciferase activity. Among this assay, a negative control was the luciferase activity of Renilla.

### 2.9. Quantitative Real-Time PCR

Total RNA of tissues or HCT116 cells was obtained by TRIzol reagent (Invitrogen, USA). The mRNA level of indicated gene was detected by utilizing a qRT-PCR system (Bio-rad, USA). U6, in addition to GAPDH, was used to be the reference of miR-378c and E2F7, respectively. Relative load of a gene was measured in the 2^−ΔΔCt^ method. The primer sequence information is provided in Table 1.

### 2.10. Western Blot

Total proteins were extracted from HCT116 cells with lysis buffer (Monad, China) and were isolated by10% SDS PAGE, which were next transferred to PVDF membrane (Thermofisher, USA). Then, the membrane was incubated with primary antibodies GAPDH (glyceraldehyde-3-phosphate dehydrogenase) (#2118, Cell Signaling Technology), Bcl-2 (#15071, Cell Signaling Technology), Bax (#5023, Cell Signaling Technology), or cleaved-Caspase-3 (#9661, Cell Signaling Technology) overnight. Subsequently, the membrane was incubated with secondary antibodies and then photographed by the Odyssey Infrared Imaging System (LI-COR, USA).

### 2.11. Statistical Analysis

All data in this study were presented in the manner of mean ± SD. Statistical difference was measured by using SPSS 19.0 system (IBM, USA) with Student's *t*-test and ANOVA. Comparisons were calculated and *P* < 0.05 was regarded to be significant statistically.

## 3. Results

### 3.1. ATRA Enhanced the Inhibitory Effect of 5-FU on Progression of HCT116 Cells and Induced Cell Apoptosis in a Concentration-Dependent Manner

To reveal the impacts of 5-FU as well as ARTA combined with 5-FU on colorectal cancer cells, HCT116 cells were employed and treated with 5-FU or 5-FU plus ATRA in indicated doses. The data illustrated that 5-FU decreased the proliferation ability of HCT116 cells and adding ATRA further downregulated cell viability compared with the control group (*P* < 0.05, Figure 1(a)). Additionally, we conducted flow cytometry and found that compared with control group, 5 *μ*M 5-FU increased the apoptosis rate of HCT116 cells and 5 *μ*M 5-FU combined with 5 *μ*M ATRA induced more cell apoptosis significantly (*P* < 0.05, Figure 1(b)). Proteins related to apoptosis were measured and the results showed that the level of Bax in addition to cleaved-Caspase-3 was upregulated while the level of Bcl2 was downregulated by 5-FU. Meanwhile, the changes were enhanced dramatically by 5-FU combined with ATRA as shown in Figure 1(c). Furthermore, treating cells with 5-FU plus ATRA exhibited the worst migration and invasion ability compared to the control group as well as the 5-FU group (*P* < 0.05, Figures 1(d) and 1(e)). Thus, ATRA enhanced the series of effects of 5-FU on HCT116 cells.

### 3.2. MiR-378c Is Downregulated in CRC and Is Positively Regulated by Treatment of 5-FU Combined with ATRA Significantly

According to ENCORI database, we discovered that the level of miR-378c was notably lower in CRC samples compared with normal samples (Figure 2(a)). In addition, we collected CRC and para-carcinoma tissues from 15 patients and conducted qRT-PCR; the results confirmed that the expression level of miR-378c was decreased dramatically in CRC tissues (*P* < 0.05, Figure 2(b)). To uncover the relationship between miR-378c and 5-FU combined with ATRA, qRT-PCR assay was applied to detect the load of miR-378c after treating with 5-FU combined with ATRA. Interestingly, we found that 5-FU increased the expression level of miR-378c and 5-FU combined with ATRA further increased the load of miR-378c in HCT116 cells (*P* < 0.05, Figure 2(c)).

### 3.3. Effects of 5-FU Combined with ATRA Are Mediated by miR-378c

To verify whether 5-FU combined with ATRA affected developments of HCT116 cells by miR-378c, we conducted MTT, transwell assay, and flow cytometry. The combined impacts of 5 *μ*M FU + 5 *μ*M ATRA (this combination possessed capacity to decrease cell viability no less than 50%) and miR-378c on progression of HCT116 were detected. The data illustrated that the effects of 5 *μ*M FU + 5 *μ*M ATRA on downregulated cell proliferation, migration in addition to invasion (*P* < 0.05, Figures 3(a)–3(c)), upregulated cell apoptosis (Figure 3(d)), and changed apoptosis-related proteins (Figure 3(e)) were partially counteracted by miR-378c inhibitor in HCT116 cells.

### 3.4. E2F7 Is the Direct Target of miR-378c

To reveal how miR-378c affected CRC, we predicated the targets of miR-378c by using ENCORI website. As presented in Figures 4(a) and 4(b), E2F7 was the direct target of miR-378c and luciferase reporter assay was used to show that the 3′UTR of E2F7 could be bound by miR-378c (*P* < 0.05). Subsequently, the expression level of E2F7 was measured after transfecting miR-378c mimic or miR-378c inhibitor. Consistently, the E2F7 expression was decreased significantly by miR-378c mimic while increased dramatically by miR-378c inhibitor in HCT116 cells (*P* < 0.05, Figure 3(c)). Thus, miR-378c was able to negatively control the expression of E2F7.

### 3.5. E2F7 Is Upregulated in CRC and Is Negatively Regulated by Treatment of 5-FU Combined with ATRA Significantly

The expression of E2F7 was suppressed significantly in CRC samples than that in normal samples according to the GEPIA database (Figure 5(a)). Consistently, the mRNA level of E2F7 in CRC tissues from 15 cases of patients was higher obviously than that in para-carcinoma tissues via using qRT-PCR experiment (*P* < 0.05, Figure 5(b)). HCT116 cells were treated with 5-FU plus ATRA, and we measured the load of E2F7 to explore the correlation between 5-FU combined with ATRA and E2F7. We discovered that 5-FU inhibited the expression level of E2F7 and its expression was further decreased by treatment of 5-FU combined with ATRA (*P* < 0.05, Figure 5(c)).

### 3.6. Effects of 5-FU Combined with ATRA Are Mediated by E2F7

To confirm that 5-FU plus ATRA inhibited the progress of CRC cells via miR-378c/E2F7 axis, we further investigated the combined effects of 5 *μ*M FU + 5 *μ*M ATRA and E2F7 on viability, migration, invasion, and apoptosis of HCT116 cells. 5 *μ*M FU + 5 *μ*M ATRA still decreased the ability of cell proliferation (Figure 6(a)), migration (Figure 6(b)), and invasion (Figure 6(c)), increased cell apoptosis rate (Figure 6(d)), and changed apoptosis-related protein expression (Figure 6(e)), which however partly were reversed by overexpressing E2F7 significantly (*P* < 0.05). Thus, E2F7 could partially counteract the inhibitory effects of 5-FU combined with E2F7 on CRC cells.

## 4. Discussion

CRC results in the second highest mortality related to cancers across the world. The reason why life expectancy of patients with CRC usually no more than 1 year is that most of them are definite diagnoses in terminal stages [24]. Chemotherapy based on 5-FU has achieved good performance in treating patients with cancer; however, resistance to 5-FU is the leading limitation for good prognosis [25]. The detailed mechanisms of resistance to 5-FU remain unclear now because of fickle biological processes [26]. Clinical trials revealed that ATRA could inhibit proliferation and promote cell apoptosis in CRC and it was then discovered to alter gene expression for exerting its functions [27]. In our study, we found that using 5-FU alone was able to decrease the viability of HCT116 cells in a dose-dependent manner, while 5-FU combined with ATRA further blocked cells to proliferate significantly. Meanwhile, combined inhibitory effects of 5-FU and ATRA also appeared in migration as well as invasion of HCT116 cells. In addition, 5-FU could promote cell apoptosis and apoptosis rate will be further increased after treatment of 5-FU plus ATRA. All above data illustrated that ATRA had the potential to enhance the anticancer effects of 5-FU and chemosensitivity of patients to 5-FU.

Previous research has reported that multiple microRNAs are associated with chemotherapy. For example, miR-100-5p is connected with cisplatin resistance of patients with lung cancer [28]. MiR-32-5p, produced in resistant cells, could trigger the PI3K/Akt signaling pathway in cancer cells [29]. MiR-145, in addition to miR-34a, serves as tumor-inhibiting factors to be associated with 5-FU resistance in CRC [30]. Notably, miRNA-378 family has been found to exert roles in cell viability, migration, invasion, and apoptosis in various cancers, including ovarian cancer [31], colon cancer [32], and so on [33, 34]. MiR-378c, one of the members of miRNA-378 family, has been reported to play a vital role in cancers such as gastric cancer and lung cancer [35, 36]. We discovered that miR-378c was downregulated in CRC according to the ENCORI database. Next, qRT-PCR was employed to confirm that the level of miR-378c was decreased in CRC tissues compared with para-carcinoma tissues. Interestingly, miR-378c could be upregulated by 5-FU alone in a concentration-dependent manner and the increase will be enhanced by adding ATRA, indicating the tight relationship between miR-378c and 5-FU combined with ATRA. Given this correlation, MTT assay, transwell assay, flow cytometry, and western blotting were conducted, and the results showed that miR-378c partially eliminated the series of effects of 5-FU combined with ATRA on CRC cells. Furthermore, E2F7 was predicted to be the direct target of miR-378c and it serves as a transcriptional suppressor to inhibit cell viability. E2F7 could play a significant role in various cancers, such as cutaneous squamous cell carcinomas [37], endometrial carcinoma [38], gallbladder cancer [39], and breast cancer cells [40]. In this study, we verified that E2F7 was regulated by miR-378c and downregulated in CRC tissues. In addition, the expression level of E2F7 was decreased by 5-FU alone and further suppressed dramatically by 5-FU combined with ATRA. Expected data illustrated that overexpression of E2F7 could partly reverse the effects of 5-FU plus ATRA on HCT116 cells, indicating that 5-FU combined with ATRA exerts its functions via miR-378c/E2F7 axis.

## 5. Conclusion

In conclusion, our study primarily revealed that ATRA enhanced the inhibitory effects of 5-FU on CRC cells through the miR-378c/E2F7 axis, which provides a type of potential therapy regimen for patients diagnosed with CRC.

## Figures and Tables

**Figure 1:** ATRA enhanced the inhibitory effects of 5-Fu on progression of HCT116 cells and induced cell apoptosis in a concentration-dependent manner. (a) Cell viability measured by MTT assay (*P* < 0.05). (b) Cell apoptosis after treating with indicated reagents. (c) The level of proteins related to cell apoptosis. (d) Migration of HCT116 cells after indicated treatment (*P* < 0.05). (e) Invasion of HCT116 cells after indicated treatment (*P* < 0.05).

**Figure 2:** MiR-378c is downregulated in CRC and is positively regulated by treatment of 5-FU combined with ATRA significantly. (a) The expression level of miR-378c in CRC according to ENCORI database. (b) The mRNA level of miR-378c in CRC tissues and para-carcinoma tissues (*N* = 15) was detected by qRT-PCR (*P* < 0.05). (c) The relationship between miR-378c and 5-FU in addition to ATRA (*P* < 0.05).

**Figure 3:** Effects of 5-FU combined with ATRA are mediated by miR-378c. (a) Cell viability after specific treatment (*P* < 0.05). (b) Migration of HC116 cells after specific treatment (*P* < 0.05). (c) Invasion of HC116 cells after specific treatment (*P* < 0.05). (d) Cell apoptosis after specific treatment. (e) The changes of proteins related to cell apoptosis.

**Figure 4:** (a) E2F7 was the direct target of miR-378c. (b) The luciferase activity of wild-type E2F7 but not mutant E2F7 was regulated by miR-378c mimic (*P* < 0.05). (c) E2F7 was downregulated by miR-378c mimic but upregulated by miR-378c inhibitor (*P* < 0.05).

**Figure 5:** E2F7 is upregulated in CRC and is negatively regulated by treatment of 5-FU combined with ATRA significantly. (a) The level of E2F7 was lower dramatically in CRC, according to GEPIA database. (b) The mRNA level of E2F7 in CRC tissues and para-carcinoma tissues was detected by qRT-PCR (*N* = 15, *P* < 0.05). (c) The relationship between E2F7 and 5-FU in addition to ATRA (*P* < 0.05).

**Figure 6:** Effects of 5-FU combined with ATRA are mediated by E2F7. (a) Cell viability after specific treatment (*P* < 0.05). (b) Migration of HC116 cells after specific treatment (*P* < 0.05). (c) Invasion of HC116 cells after specific treatment (*P* < 0.05). (d) Cell apoptosis after specific treatment. (e) The changes of proteins related to cell apoptosis.

**Table 1:** The sequence of primer.

Gene	RT-PCT primer
MiR-378c	Forward: 5ʹ GAGGCCATCACTGGACTTGG-3ʹ
	Reverse: 5ʹ-GAGGCACTCACCACCTTCAAA-3ʹ
U6	Forward: 5ʹ CTCGCTTCGGCAGCACA-3ʹ
	Reverse: 5ʹ-AACGCTTCACGAATTTGCGT-3ʹ
E2F7	Forward: 5ʹ-AATGCAGTGGTTGTTTCTGT-3ʹ
	Reverse: 5ʹ-TGCCATTGCTTCTTCACTAC-3ʹ
GAPDH	Forward: 5ʹ-GGGAAACTGTGGCGTGAT-3ʹ
	Reverse: 5ʹ-GAGTGGGTGTCGCTGTTGA -3ʹ

## Data Availability

The data used to support the findings of this study are included within the article.
